The article "Gene expression analysis in response to osmotic stimuli in the intervertebral disc with DNA microarray" was retracted in 2015. Reasons: compromised peer review; ethical violations by an institution or third party; concerns about the results or conclusions.

# Gene expression analysis in response to osmotic stimuli in the intervertebral disc with DNA microarray

**DOI:** 10.1186/2047-783X-18-62

**Published:** 2013-12-27

**Authors:** Wenzhi Zhang, Xu Li, Xifu Shang, Qichun Zhao, Yefeng Hu, Xiang Xu, Rui He, Liqun Duan, Feng Zhang

**Affiliations:** 1 Department of Orthopaedics, Anhui Provincial Hospital, No. 17, Road Lujiang, Hefei 230001, China

**Keywords:** Intervertebral disc, Top-scoring pair, Osmotic pressure, Osmotic stimuli

## Abstract

**Background:**

Intervertebral disc (IVD) cells experience a broad range of physicochemical stimuli under physiologic conditions, including alterations in their osmotic environment. At present, the molecular mechanisms underlying osmotic regulation in IVD cells are poorly understood. This study aims to screen genes affected by changes in osmotic pressure in cells of subjects aged 29 to 63 years old, with top-scoring pair (TSP) method.

**Methods:**

Gene expression data set GSE1648 was downloaded from Gene Expression Omnibus database, including four hyper-osmotic stimuli samples, four iso-osmotic stimuli samples, and three hypo-osmotic stimuli samples. A novel, simple method, referred to as the TSP, was used in this study. Through this method, there was no need to perform data normalization and transformation before data analysis.

**Results:**

A total of five pairs of genes ((*CYP2A6*, *FNTB*), (*PRPF8*, *TARDBP*), (*RPS5*, *OAZ1*), (*SLC25A3*, *NPM1*) and (*CBX3*, *SRSF9*)) were selected based on the TSP method. We inferred that all these genes might play important roles in response to osmotic stimuli and age in IVD cells. Additionally, hyper-osmotic and iso-osmotic stimuli conditions were adverse factors for IVD cells.

**Conclusions:**

We anticipate that our results will provide new thoughts and methods for the study of IVD disease.

## Background

Intervertebral disc (IVD) disease is a frequent surgical disease characterized by a series of deleterious changes in cellularity that lead to loss of extracellular matrix structure, altered biomechanical loading, and symptomatic pain [1]. Although studies of biological therapeutics for IVD disease have been ongoing over a decade, few treatments have progressed to clinical testing and none is current commercially available [2-4]. This may be, primarily, due to a limited understanding of disease etiology. Therefore, further work is needed to explore its pathogenesis from early to later stages.

The IVD, an avascular and lymphatic tissue, is composed of different zones, including the annulus fibrosus, the nucleus pulposus, and the transition zone [5]. The IVD cells can secrete a complex extracellular matrix containing lots of water and negatively charged proteoglycans, which confer a net negative charge on the tissue and give the tissue a higher extracellular osmolarity than other tissues [6,7]. Previous studies have shown that IVD cells respond strongly to changes in the osmotic environment by altering mRNA expression [8]. In particular, the genes encoding proteins related to ion transport, cytoskeletal organization, growth factors, and cytokines have been demonstrated to show different regulation response to osmotic conditions in IVD cells [6,9,10]. Meanwhile, both hyper- and hypo-osmotic conditions can induce changes of cell volume and calcium signaling in IVD cells [11,12]. However, the molecular mechanisms involved in the response of IVD cells to osmotic pressure are still not clearly understood.

In the present study, gene expression profile data of IVD cells exposed to iso-osmotic, hyper-osmotic, and hypo-osmotic conditions were downloaded. Top scoring pair (TSP) is a novel, simple statistical method that can classify gene pairs into relevant classes based on their scores [13-15]. In this study, the TSP method was used to screen the pairs of differentially expressed genes in different osmotic stimuli conditions. Our findings might shed new light on the molecular mechanisms of human IVD disease.

## Methods

### Gene expression data

Expression profiling of GSE1648 [9] was downloaded from Gene Expression Omnibus (GEO, http://www.ncbi.nlm.nih.gov/geo/), based on GPL96 [HG-U133A] Affymetrix Human Genome U133A Array. A total of 11 human IVD tissue samples were collected, including four hyper-osmotic stimuli samples (ages: 63, 62, 50, and 29, respectively), four iso-osmotic stimuli samples (ages: 63, 62, 50, and 29, respectively) and three hypo-osmotic stimuli samples (ages: 63, 50, and 29, respectively).

### Top-Scoring Pair (TSP)

Recently, gene pair response to environmental changes has been assessed using the TSP method, which is based on pair-wise comparisons of gene expression values within each tissue microarray [16]. Distinction between two classes depended on the gene pairs with the highest ranking value (called “score”). In the current study, the higher score of the gene pairs indicated the stronger correlation between the expression values of gene-pairs and tissues.

### Algorithm overview of the TSP method

Detailed information about the TSP method was described by Geman et al. [16]. Here, we give a brief and intuitive description of this method. A gene expression profile consists of G genes and N samples (i.e., hypo-osmotic) participating in the training micro-array dataset. The data is represented as a G × N matrix, in which the expression value of g^th^ gene from the n^th^ sample is denoted as “Xgn”. Each column represents a gene expression profile of G genes and each row represents observations of a particular gene over N samples. Each sample has a class label of either 1 or 2. For the simplicity of calculations, it is assumed that there are only two classes, and we assume that samples 1 to N1 (N1 < N) are labeled as class 1 (e.g., hyper-osmotic) and samples (N1 + 1) to N are labeled as class 2 (e.g., iso-osmotic). For each pair of genes (i, j), two probabilities are calculated as *pij* (1) and *pij* (2):

$$\begin{array}{l} p_{\mathrm{ij}}\left(1\right)=\frac{1}{N_{1}}\sum_{n=1}^{N_{1}}I_{\left(X_{\mathrm{in}}<X_{\mathrm{jn}}\right)},\\ \;p_{\mathrm{ij}}\left(2\right)=\frac{1}{N-N_{1}}\sum_{n=N_{1}+1}^{N}I_{\left(X_{\mathrm{in}}<X_{\mathrm{jn}}\right)} \end{array}$$

*I*_(Xin < Xjn)_ is the indicator function defined as:

$$I_{\left(\mathrm{Xin}<\mathrm{Xjn}\right)}=\left[{}_{0,\;\mathrm{if}\;\left(X_{\mathrm{in}}>X_{\mathrm{jn}}\right)}^{1,\;\mathrm{if}\;\left(X_{\mathrm{in}}<X_{\mathrm{jn}}\right)}\right)n=1,2\ldots N.$$

TSP is a rank-based method, so for each pair of genes (i, j), the “score” denoted as Δ_ij_ is calculated as follows:

$$\Delta_{\mathrm{ij}}=\left|p_{\mathrm{ij}}\left(1\right)-p_{\mathrm{ij}}\left(2\right)\right|$$

In other words, *pij* (1) (or *pij* (2), respectively) is the estimated probability of observing X_i_ less than X_j_ in class 1 (or class 2). Δ_ij_ is the absolute value of the difference between *pij* (1) and *pij* (2) and represents the difference of pairs of genes (i, j) between class 1 and class 2. In this study, the larger the Δ_ij_ (close to 1), the greater the difference of pairs of genes (i, j) between class 1 and class 2, indicating that pairs of genes (i, j) may be related to the tissues. Meanwhile, Δ_ij_ >0.6 was set as cut-off criteria. In addition, the TSP method focuses on gene-pair (i, j) matching between two classes.

In the present study, we divided the samples into three groups: hyper-osmotic vs. hypo-osmotic group, hyper-osmotic vs. iso-osmotic group, and iso-osmotic vs. hypo-osmotic group.

### Osmotic pressure*,* age, and related genes

To reduce the false positive rate, we analyzed the potential relationship between age and osmotic pressure based on the Δ_ij_ score. All pairs of genes with the largest score (Δ_ij_ = 0.75) and that repeatedly appeared in the three groups (≥2) were selected. Then, the expression level of gene pairs from hyper-osmotic stimuli samples with the ages of 63, 62, 50, and 29 was analyzed, respectively, as was the expression of iso-osmotic stimuli samples (ages: 63, 62, 50, and 29, respectively) and hypo-osmotic stimuli samples (ages: 63, 50, and 29, respectively), in order to present a tendency of gene expression along with age.

## Results

### Osmotic pressure and related genes

Based on the TSP method, a total of 65 gene pairs were selected from the three groups, including 34 gene pairs in the hyper-osmotic vs. hypo-osmotic group (Table 1), 7 in hyper-osmotic vs. iso-osmotic group (Table 2), and 24 in iso-osmotic vs. hypo-osmotic group (Table 3). For the hyper-osmotic vs. hypo-osmotic group (Table 1), a total of 34 gene pairs were obtained with Δ_ij_ >0.6, including a gene pair with Δ_ij_ = 1, 11 gene pairs with Δ_ij_ = 0.75, and 22 gene pairs with Δij = 0.666667. For the hyper-osmotic vs. iso-osmotic group (Table 2), a total of 7 gene pairs were obtained with Δ_ij_ >0.6 and the Δ_ij_ were all = 0.75. For the iso-osmotic vs. hypo-osmotic group (Table 3), a total of 24 gene pairs were obtained at Δ_ij_ >0.6, including a gene pair with Δ_ij_ = 1, 7 with Δ_ij_ = 0.75, and 16 with Δ_ij_ = 0.666667.

**Table 1:** The screening results of pairs of genes in hyper-osmotic vs. hypo-osmotic group based on the top-scoring pair method

**First ID**	**Second ID**	***pij*** **(1)**	***pij*** **(2)**	Δ_**ij**_
1	21	0	0.666667	0.666667
1	35	0	0.666667	0.666667
5	10	1	0.333333	0.666667
8	18	0.25	1	0.75
9	10	1	0.333333	0.666667
13	17	0.25	1	0.75
23	31	0.75	0	0.75
23	85	1	0.333333	0.666667
29	60	0.25	1	0.75
29	62	0	0.666667	0.666667
29	76	0	0.666667	0.666667
30	78	0	0.666667	0.666667
31	85	1	0.333333	0.666667
32	49	1	0.333333	0.666667
33	46	0.25	1	0.75
34	85	1	0.333333	0.666667
37	38	0.25	1	0.75
40	80	0.75	0	0.75
45	98	0.75	0	0.75
51	85	1	0.333333	0.666667
57	85	1	0.333333	0.666667
58	65	0.75	0	0.75
58	88	1	0.333333	0.666667
61	88	1	0.333333	0.666667
62	88	0.75	0	0.75
62	99	1	0.333333	0.666667
63	94	0	0.666667	0.666667
65	93	1	0.333333	0.666667
67	69	1	0.333333	0.666667
68	74	0	0.666667	0.666667
72	75	1	0.333333	0.666667
76	88	0.75	0	0.75
76	99	1	0	1
80	86	0	0.666667	0.666667

Footnote: First ID represents genes in intervertebral disc cells with hyper-osmotic stimuli. Second ID represents genes in intervertebral disc cells with hypo-osmotic stimuli.

**Table 2:** The screening results of pairs of genes in hyper-osmotic vs. iso-osmotic group based on the top-scoring pair method

**First ID**	**Second ID**	***pij*** **(1)**	***pij*** **(2)**	Δ_**ij**_
21	41	0	0.75	0.75
37	51	0.75	0	0.75
37	85	1	0.25	0.75
51	84	0	0.75	0.75
58	65	0.75	0	0.75
58	68	0.75	0	0.75
71	92	0.75	0	0.75

Footnote: First ID represents genes in intervertebral disc cells with hyper-osmotic stimuli conditions. Second ID represents genes in intervertebral disc cells with iso-osmotic stimuli conditions.

**Table 3:** The screening results of pairs of genes in iso-osmotic vs. hypo-osmotic group based on the top-scoring pair method

**First ID**	**Second ID**	***pij*** **(1)**	***pij*** **(2)**	Δ_**ij**_
2	8	1	0.333333	0.666667
9	10	1	0.333333	0.666667
13	17	0.25	1	0.75
19	41	1	0.333333	0.666667
21	41	0.75	0	0.75
22	54	1	0.333333	0.666667
23	85	1	0.333333	0.666667
26	36	1	0.333333	0.666667
29	62	0	0.666667	0.666667
30	78	0	0.666667	0.666667
31	84	1	0.333333	0.666667
31	85	1	0.333333	0.666667
34	45	0	0.666667	0.666667
37	45	0	1	1
37	51	0	0.666667	0.666667
40	84	1	0.333333	0.666667
43	45	0	0.666667	0.666667
45	98	0.75	0	0.75
49	66	0	0.666667	0.666667
49	96	0.25	1	0.75
51	84	0.75	0	0.75
58	76	0.25	1	0.75
70	71	1	0.333333	0.666667
71	97	0.25	1	0.75

Footnote: First ID represents genes in intervertebral disc cells with iso-osmotic stimuli. Second ID represents genes in intervertebral disc cells with hyper-osmotic stimuli.

### Age and related genes

As shown in Table 4, a total of five gene pairs might have potential relationships between age and osmotic pressure, including (*CYP2A6*, *FNTB*), (*PRPF8*, *TARDBP*), (*RPS5*, *OAZ1*), (*SLC25A3*, *NPM1*), and (*CBX3*, *SRSF9*).

**Table 4:** The screening result of osmotic stimuli and age in intervertebral disc cells

**Term**	**H63**	**H62**	**H50**	**H29**	**I63**	**I62**	**I50**	**I29**	**L63**	**L50**	**L29**
**Gene name**											
CYP2A6	295.0	254.8	254.1	313.8	252.6	227.8	276.0	235.8	198.4	160.7	202.9
FNTB	203.3	125.5	173.0	345.8	152.3	189.2	145.8	284.6	215.8	252.5	224.7
PRPF8	2524.9	1718.9	1835.8	1770.8	2300.4	1583.1	1114.4	1858.9	2568.2	1633.9	1696.9
TARDBP	661.2	1376.6	1318.0	1676.1	1027.4	1585.4	1149.8	1907.7	925.3	873.1	1198.6
RPS5	12991.9	7421.0	7272.1	9049.5	9314.9	7835.8	7309.5	8288.9	11266.1	9597.2	9900.7
OAZ1	7997.4	7819.5	7895.4	9254.5	7333.8	8252.4	7572.8	9327.2	8224.7	9151.1	9733.9
SLC25A3	10720.2	9369.4	7140.9	9115.2	8745.7	9064.5	6827.8	8444.5	10780.3	7778.3	9579.1
NPM1	9818.2	8637.1	5232.9	6995.0	10720.1	9126.9	7056.0	8196.5	9834.5	6465.2	8610.2
CBX3	1652.5	1798.9	2067.2	2568.6	2040.8	2078.3	2900.1	2671.4	1992.7	2375.8	2444.9
SRSF9	2073.6	2120.3	2124.0	1361.8	2004.9	1826.6	2576.8	1757.2	1797.8	2304.2	1917.4

Footnote: (1) H, I, L represent hyper-osmotic stimuli, iso-osmotic stimuli, and hypo-osmotic stimuli, respectively. (2) The number of H/I/L represents the age. (3) The data in the table is the expression value of each gene in different osmotic stimuli conditions and ages.

For the (*CYP2A6*, *FNTB*) pair, at the ages of 50–63, the gene expression value of *CYP2A6* was more than that of *FNTB* in both hyper-osmotic and iso-osmotic stimuli samples, and the situation was reversed in the hypo-osmotic stimuli samples. However, at age 29, the gene expression value of *CYP2A6* was always less than that of *FNTB*.

For the (*PRPF8*, *TARDBP*) pair, at the ages of 29–63, the expression value of *PRPF8* was more than that of *TARDBP* in both hyper-osmotic and hypo-osmotic stimuli samples. In iso-osmotic stimuli samples, the expression level of *PRPF8* was similar to that of *TARDBP*.

For the (*RPS5*, *OAZ1*) pair, at the ages of 29–62, the expression level of *RPS5* was always lower than that of *OAZ1* in both hyper-osmotic and iso-osmotic stimuli samples; however, the situation was reversed at the age of 63. Meanwhile, in hypo-osmotic stimuli samples, the expression level of *RPS5* was always higher than that of *OAZ1*.

For the (*SLC25A3*, *NPM1*) pair, the gene expression values were reversed in different osmotic pressure. At the ages of 29–63, the gene expression value of *SLC25A3* was always larger than that of *NPM1* in both hyper-osmotic and hypo-osmotic stimuli samples. Meanwhile, the situation was reversed in the iso-osmotic stimuli samples except at the age of 29.

For the (*CBX3*, *SRSF9*) pair, at the ages of 29–63, the gene expression value of *CBX3* was always larger than that of *SRSF9* in both iso-osmotic and hypo-osmotic stimuli samples. However, in the hyper-osmotic stimuli samples, the gene expression value of *CBX3* was more than that of *SRSF9* at the age of 29 and the situation was reversed at the age of 50–63.

All these results indicated that the expression level of these gene pairs ((*CYP2A6*, *FNTB*), (*PRPF8*, *TARDBP*), (*RPS5*, *OAZ1*), (*SLC25A3*, *NPM1*) and (*CBX3*, *SRSF9*)) at different osmotic pressures did not change at an early age, but was reversed in old age.

## Discussion

In the current study, it was shown that five gene pairs might be involved in the potential interaction between osmotic pressure and age, (*CYP2A6*, *FNTB*), (*PRPF8*, *TARDBP*), (*RPS5*, *OAZ1*), (*SLC25A3*, *NPM1*) and (*CBX3*, *SRSF9*). The expression level of the five gene pairs was not influenced by the changes in osmotic pressure at an early age, but was influenced in old age. These results suggest that these gene pairs may be associated with the regulation mechanism of the senescence of IVD tissue and that the IVD tissue of aged people may be sensitive to the changes in osmotic pressure as a result of wearing and aging.

Cytochrome P450 2A6 (*CYP2A6*) is a member of the cytochrome P450 (*CYP*) mixed-function oxidase system, which is involved in the oxidation of nicotine and cotinine, and the metabolism of several pharmaceuticals, carcinogens, and coumarin-type alkaloids [17-20]. It has been reported that *CYP* may be involved in the activation of caspase 12 that acts directly on the cell and mediates the effector caspase 3 resulting in apoptosis [21]. The *FNTB* gene encodes the protein farnesyltransferase subunit beta which plays an important role in protein farnesylation, regulation of cell proliferation, microtubule complex, and protein farnesyltransferase complex [22,23]. In addition, we found the expression value of the *FNTB* gene was less than that of the *CYP2A6* gene both in hyper-osmotic and iso-osmotic conditions at an old age. Therefore, we inferred that the *FNTB* gene and the *CYP2A6* gene may play opposite roles in IVD cells and that the hyper-osmotic conditions at an old age may be a negative factor for IVD cells.

*PRPF8*, together with *PRPF3* and *PRFP31*, encodes splicing factors and accounts for approximately 15% of families with autosomal dominant retinitis pigmentosa in the UK [24]. No report has revealed an association between the expression of *PRPF8* and IVD. Meanwhile, *TARDBP*, encoding TAR-DNA binding protein (also known as TDP-43 proteins), is one of the principal genes responsible for the adult onset form of amyotrophic lateral sclerosis (ALS), displaying a TDP-43 positive skein-like inclusions in the anterior horn of the spinal cord and inferior olive [25]. It has been suggested that the calpain-dependent cleavage of TDP-43 plays a crucial role in ALS [26]. In the present study, the expression level of *PRPF8* was larger than that of *TARDBP* in both hyper-osmotic and hypo-osmotic stimuli samples, especially at an old age. These results suggested a greater susceptibility of *PRPF8* than *TARDBP* to osmotic stimuli response.

*RPS5* encodes ribosomal protein s5 and has been suggested as one of the most stable reference genes for qPCR analysis of degenerated nucleus pulposus tissue (a fundamental component of IVD degeneration) in dogs [27]. *OAZ1* encodes ornithine decarboxylase antizyme 1, a negative regulator of cellular polyamines, and has been suggested as a potential genetic marker of vascular events [28]. To date, the contribution of *OAZ1* to IVD has not been explored. In our study, the different expression of *RPS5* and *OAZ1* genes in hyper-osmotic and hypo-osmotic stimuli samples suggested different response functions to osmotic conditions in IVD cells.

The *SLC25A3* gene encodes a phosphate carrier protein (also named phosphate transport protein, PTP) which is a member of the solute carrier (SLC) family and is located in mitochondria [29]. PTP catalyzes the transport of phosphate groups from the cytosol to the mitochondrial matrix, either by proton co-transport or in exchange for hydroxyl ions [30]. To date, there is no direct evidence of *SLC25A3* ever regulating osmotic pressure, however, it has been reported that the expressions of *SLC21A12*, *SLC5A3*, and *SLC16A6* are regulated by osmotic conditions in IVD cells, which is consistent with our results [31]. Meanwhile, nucleophosmin (NPM) (also known as nucleolar phosphoprotein B23 or numatrin) is encoded by the *NPM1* gene in humans [32,33]. To date, there is no report revealing the contribution of NPM to IVD. NPM may be involved in diverse biological functions, such as ribosome biogenesis and transport, genomic stability and DNA repair, endoribonuclease activity, and centrosome duplication during the cell cycle [34-37]. As a result, we inferred that the changes of expression level of *NPM* may be used to explain the changes of IVD cells in sensitivity to osmotic pressure and the phenomenon of disc degeneration in old age [38,39]. In our study, we found the expression level of the *SLC25A3* gene to be less than the *NPM1* gene only in iso-stimuli conditions in old age. Therefore, we inferred that iso-stimuli conditions might be an adverse factor for IVD cells.

Chromobox protein homolog 3 (HP1 gamma) is encoded by the *CBX3* gene and is involved in chromatin remodeling, DNA-dependent transcription, and negative regulation of transcription [40,41]. Furthermore, it has been reported that HP1 plays an important role in cell survival, by supporting cell proliferation [33]. Meanwhile, serine/arginine rich splicing factor 9 (*SRSF9*), a member of the serine/arginine-rich protein family, is involved in alternative pre-mRNA splicing and plays a critical role in the regulation of apoptosis by splicing apoptosis-related genes [42,43]. Therefore, these studies may explain the lower expression level of the *CBX3* gene compared to that of the *SRSF9* gene in our study.

To summarize, we inferred that hyper-osmotic and iso-osmotic conditions were adverse environmental factors for IVD cells, which was consistent with a previous study showing that IVD tissues have a higher extracellular osmolality than most other tissues [6,7]. However, it should be pointed out that several limitations were present in our study. The human IVD tissue samples were collected from patients aged 63, 62, 50, and 29 years old. The number of gene expression profiles was limited. Additionally, samples with a wider age range are needed to further analyze and confirm our inferences. Further, no computational procedure is perfect; as a result, potential candidates might be missed. In our study, only five pairs were identified; however, other important gene pairs might also be elucidated through other analysis methods and different samples.

## Conclusions

In conclusion, we explored the molecular mechanism of the different responses of IVD cells in hyper-osmotic, iso-osmotic, and hypo-osmotic conditions. Finally, five gene pairs ((*CYP2A6*, *FNTB*), (*PRPF8*, *TARDBP*), (*RPS5*, *OAZ1*), (*SLC25A3*, *NPM1*) and (*CBX3*, *SRSF9*)) were selected based on the TSP method. Our results indicated that the expression level of these genes was reversed in old age in different osmotic stimuli conditions, but the expression level of these genes was not affected at an early age. We believe our results may provide new information on the molecular mechanisms of IVD disease.

## Abbreviations

ALS: Amyotrophic lateral sclerosis; GEO: Gene expression omnibus; HP1: Chromobox protein homolog 3; IVD: Intervertebral disc; NPM: Nucleophosmin; PTP: Phosphate transport protein; SLC: Solute carrier; SRSF9: Serine/arginine rich splicing factor 9; TSP: Top-scoring pair.

## Competing interests

The authors declare that there are no any conflicts of interest.

## Authors’ contributions

WZZ, XL and XFS conceived and designed the article, collected and analyzed the data and wrote the paper. QCZ, YFH and XX participated in analyzing the data and drafted the manuscript. RH, LQD and FZ analyzed the data. All authors read and approved the final manuscript.
